The article "Effect of Psychological Nursing Intervention on Abnormal-Induced Labor of Fetus during Puerperium: Study on the Effects of Anxiety, Depression, and Life Events" was published in 2022. Journal: Comput Math Methods Med.

# Effect of Psychological Nursing Intervention on Abnormal-Induced Labor of Fetus during Puerperium: Study on the Effects of Anxiety, Depression, and Life Events

**DOI:** 10.1155/2022/6206851

**Published:** 2022-08-23

**Authors:** Yanjuan He, Huiwen He, Cai Tang

**Affiliations:** ^1^Department of Obstetrics, Changsha Hospital for Maternal and Child Health Care, Changsha 410000, China; ^2^Department of Neurology, Hunan Children's Hospital, Changsha, Hunan 410000, China; ^3^Department of Gynecology, Hunan Provincial People's Hospital (The First Affiliated Hospital of Hunan Normal University), Changsha, Hunan 410000, China

## Abstract

**Objective:**

To study the effects of psychological nursing intervention on anxiety, depression, and life events in puerperal women with fetal abnormalities.

**Methods:**

From January 2020 to January 2022, eighty women with abnormal fetal induction and puerperium-treated were selected in our hospital as the subjects. The research group (*n* = 40) and control group (*n* = 40) were arbitrarily selected from 80 women with abnormal fetal induction and puerperium. The research group was given psychological nursing intervention based on routine nursing, and the control cases were given routine nursing. The scores of Generalized Anxiety Scale (GAD-7), Patient Health Questionnaire (PHQ-9), Event Impact Scale (IES-R), Life Events Scale (LES), and Newcastle Nursing Satisfaction Scale (NSNS) were studied before nursing and 4 weeks after discharge.

**Results:**

Four weeks after discharge, the score of GAD-7 in the research group was lower, and the difference was statistically significant (*P* < 0.05). The score of PHQ-9 in the research group was lower, and the difference was statistically significant (*P* < 0.05). The IES-R score of the research group was lower, and the difference was statistically significant (*P* < 0.05). The LES score of the research group was lower, and the difference was statistically significant (*P* < 0.05). And the NSNS score of the research group was higher, and the difference was statistically significant (*P* < 0.05).

**Conclusion:**

The value of psychological care interventions in women with abnormally induced labor is more remarkable, contributing to the reduction of anxiety and depression and increasing the satisfaction of care for women with abnormally induced labor.

## 1. Introduction

Fetal abnormalities include congenital malformations and stillbirths [1]. Fetal congenital malformation refers to the abnormal development of fetal morphology, structure, and physiological function caused by various internal and external factors in the process of embryonic development [2]. Stillbirth refers to fetal death in the womb after 20 weeks of pregnancy [3]. The progress of prenatal diagnosis technology has greatly improved the diagnosis rate of fetal developmental abnormalities. The current intrauterine treatment techniques are still very limited. Once the fetus is diagnosed with serious developmental abnormalities, we must face the cruel reality and fierce emotional struggle to terminate the pregnancy [4, 5]. Termination of pregnancy is necessary when fetal malformations are detected during pregnancy. This is a strong psychological shock and emotional blow to the pregnant woman and can bring about devastating psychosocial problems [6]. Previous studies have shown that such events can cause posttraumatic stress disorder (PTSD) in women with abnormal fetal induction of labor, as well as strong negative emotions such as anxiety, depression, helplessness, fear, and dissatisfaction [7, 8]. In addition, the symptoms of PTSD and depression caused by abnormal-induced labor indicated a persistent pattern, which persisted for 2-7 years after induced labor [9]. In recent years, a number of studies have found that women have negative psychological experiences after the traumatic event of an abnormal fetal induction. The psychological torment of women with abnormal fetal induction is so severe that they may even be suicidal [10, 11]. From placenta delivery to the maternal body organs (except breast) to restore to the normal nonpregnant state of a period (generally 6 weeks) is called puerperal period [2]. Puerperium is a critical period for the physical and psychological recovery of pregnant women. Previous studies have shown that postpartum 3-7 days is the peak period of anxiety and depression in puerperal women [12, 13]. Most women with induced labor have a short hospitalization time and can be discharged from hospital 2-3 days after induced labor. There are few social support resources available during puerperal period after discharge. Physical and mental rehabilitation and nursing are weak links at this stage. Psychological nursing intervention has become a widely concerned field of maternal and obstetrical health care in China. A few studies have shown that psychological nursing intervention model can fully meet the health needs of puerperal women, reduce the occurrence of postpartum depression, increase self-care ability, successfully complete the role transformation, and promote the physical rehabilitation of parturients [14, 15]. Therefore, this paper formulated the intervention program for the puerperal psychology of women with fetal abnormal-induced labor and verified the effects of the intervention program on puerperal anxiety, depression, and life events.

## 2. Patients and Methods

### 2.1. General Information

During January 2020 to January 2022, eighty women with abnormal fetal induction and puerperium-treated were selected in our hospital as the subjects. The research group (*n* = 40) and control group (*n* = 40) were arbitrarily selected from 80 women with abnormal fetal induction and puerperium. In the former group, the age distribution ranged from 29 to 38 years old with an average of (31.48 ± 2.16) years. The gestational age was between 14 and 35 weeks with an average of (25.74 ± 3.12) weeks. In the latter group, the age distribution was from 28 to 39 years old with an average of (31.15 ± 2.33) years. The gestational weeks were between 14 and 34 weeks with an average of (25.69 ± 3.19) weeks. Inclusion criteria were as follows: (1) pregnant women were diagnosed as fetal malformations or stillbirths by prenatal diagnosis; (2) hospitalized for induced labor, the gestational week at the time of induced labor was ≥14 weeks; (3) the individual had not received psychotherapy or counseling recently; and (4) a pregnant woman and her family are voluntarily participating in this study and signed an informed consent form. Exclusion criteria were as follows: (1) previous patients with severe mental disorders (including schizophrenia, mania, severe depression, anxiety disorders and other psychotic disorders), history of mental illness, and unable to complete; (2) people with hearing and expression disorders; (3) those who could not understand the contents of the questionnaire, such as illiteracy and low education level; (4) previous history of fetal malformation and stillbirth; and (5) pregnancy termination was performed due to other reasons.

### 2.2. Treatment Methods

#### 2.2.1. Technical Route

The technical route of this study was shown in Figure 1.

#### 2.2.2. Intervention Program

The protocol for the control group was for patients to receive routine diagnosis, treatment, and care. Routine admission education was then given, and invitations to join the control group's microgroup were made. The researcher established a good nurse-patient relationship with the subjects on the day of admission and conducted admission health education and discharge education. Interaction and feedback were always maintained with the mother via WeChat during the puerperium. Follow-up visits were made two weeks after discharge and 42 days after delivery to remind and inform women about the hospital review and the process. The whole intervention consists of 4 weeks.

The scheme of the research group is as follows: psychological nursing intervention was carried out on the basis of routine nursing. The researchers established a good nurse-patient relationship with the subjects on the day of admission. The woman's anxiety and depression were assessed. Patients expressing their current worries and concerns were encouraged, and targeted admission health education (e.g., basic concepts and diagnosis of fetal abnormalities, methods and precautions for termination of pregnancy, and family support education) was given. In addition, the individualized instruction time was 30-50 min. One-to-one postnatal health education (what to do after termination of pregnancy) for the subject at the bedside 24 hours was performed after induction of labor. Yoga instruction and evaluation of the subject's practice were needed for 30-40 min. Yoga was required to practice yoga once a day before discharge. Pregnancy-related knowledge and health education were enhanced. Similar success stories of women having second pregnancies were shared to guide women to understand the disease properly to reduce guilt and alleviate negative emotions. The subjects' yoga practice was evaluated and guides them to write a record of the intervention topics. After discharge, the patients were intervened for 4 weeks through the online WeChat platform with the theme course 30 min every week. Pregnancy and childbirth science was regularly promoted through the online WeChat platform, which provided an opportunity for mothers and their spouses to exchange information and emotions. Invite pregnant women who have had another successful pregnancy to enhance their faith in another successful pregnancy. The content of family support is reinforced, and patients give positive feedback to their families through practical actions expressing gratitude. The patients were guided to explore available social support resources and write weekly intervention themes. During the intervention, pregnant women were urged to complete their homework via WeChat to improve intervention compliance. The intervention should be timed to avoid the subject's treatment and daily care time. The whole intervention process included 4 weeks.

### 2.3. Observation Indicators

1. The scores of GAD-7 before nursing and 4 weeks after discharge: the GAD-7 scale [16] was used to evaluate the anxiety state of parturients with fetal abnormality-induced labor. There were 7 items in the scale, and each item was scored according to 0-3. The total score of the scale was 0-21, including 0-4 as no anxiety, 5-9 as mild anxiety, 10-14 as moderate anxiety, and ≥15 as severe anxiety. Cronbach's *α* coefficient of the scale was 0.92 [17]
2. The scores of PHQ-9 before nursing and 4 weeks after discharge: the PHQ-9 scale was used to evaluate the depression status of parturients with fetal abnormality-induced labor [18]. There were 9 items in the scale. The total score of the scale was 0-27. Depression levels increase as the score increases. There was no depression in score that ranges 0-4, mild depression was 5-8, moderate depression was 9-10, severe depression was 15-19, and extremely severe depression was 20-27. Cronbach's *α* coefficient of the scale was 0.89 [19]
3. The scores of IES-R before nursing and 4 weeks after discharge: the revised version of the IES-R scale was a commonly used tool to assess the performance and severity of posttraumatic stress response in the world [20]. A total of 22 items were divided into three dimensions, including intrusion, escape, and arousal, including 8 entries in intrusion dimension (1, 2, 3, 6, 9, 14, 16, 20), 8 items in escape dimension (5, 7, 8, 11, 12, 13, 17, 22), and 6 entries in arousal dimension (4, 10, 15, 18, 19, 21). Using the 5-level scoring method, from “no impact” to “especially many” represented the “0 ~ 4” score with a total score of 0 ~ 88. Foreign studies have found that people with a total score of more than 19 points were regarded as the standard of clinical attention [21]. The scale had good reliability and validity, and Cronbach's *α* coefficient was 0.89 [22]
4. The scores of LES before nursing and 4 weeks after discharge: the LES [23] included family life (28 items), work and study (13 items), and social and other aspects (7 items). There were 2 blank items, and the degree of influence was divided into 5 grades. 0, 1, 2, 3, and 4 points were scored from no influence to extremely serious influence
5. The scores of NSNS before nursing and 4 weeks after discharge: the total score of NSNS scale ranged from 0 to 95 [24]. Each item was evaluated with a score of 1 to 5, of which 1: very displeased, 2: displeased, 3: general satisfaction, 4: pleased, and 5: very pleased

### 2.4. Statistical Analysis

SPSS23.0 statistical software was adopted to process the data. The measurement data were presented as ($\bar{x}\pm s$). The group design *t*-test was adopted for the comparison, and the analysis of variance was adopted for the comparison between multiple groups. Dunnett's *t*-test was adopted for comparison with the control group. The counting data were presented in the number of cases and the percentage, *χ*^2^ test was adopted for comparison between groups, and bilateral test was employed for all statistical tests.

## 3. Results

### 3.1. Comparison of General Data

There exhibited no remarkable difference in demographic data such as age, gestational week, education level, bad pregnancy history, with or without children, pregnancy type, and fetal abnormality type (*P* > 0.05), as shown in Table 1.

### 3.2. The Scores of GAD-7 Scale before Nursing and 4 Weeks after Discharge

Before nursing, there exhibited no remarkable difference in the score of the GAD-7 scale (*P* > 0.05). Four weeks after discharge, the score of GAD-7 in the research group was lower, and the difference was statistically significant (*P* < 0.05), as shown in Table 2.

### 3.3. The Scores of PHQ-9 before Nursing and 4 Weeks after Discharge

Before nursing, there exhibited no remarkable difference in the score of the PHQ-9 scale (*P* > 0.05). Four weeks after discharge, the score of PHQ-9 in the research group was lower, and the difference was statistically significant (*P* < 0.05), as shown in Table 3.

### 3.4. The IES-R Score of Two Groups before Nursing and 4 Weeks after Discharge

Before nursing, there exhibited no remarkable difference in the score of the IES-R scale (*P* > 0.05). Four weeks after discharge, the IES-R score of the research group was lower, and the difference was statistically significant (*P* < 0.05), as shown in Table 4.

### 3.5. The Score of LES Scale before Nursing and 4 Weeks after Discharge

Before nursing, there exhibited no remarkable difference in the score of the LES scale (*P* > 0.05). Four weeks after discharge, the LES score of the research group was lower, and the difference was statistically significant (*P* < 0.05), as shown in Table 5.

### 3.6. NSNS Scale Score before Nursing and 4 Weeks after Discharge

Before nursing, there exhibited no remarkable difference in the score of the NSNS scale (*P* > 0.05). Four weeks after discharge, the NSNS score of the research group was higher, and the difference was statistically significant (*P* < 0.05), as shown in Table 6.

## 4. Discussion

China's “second child” policy has led to a sharp increase in the number of elderly pregnant women. The development of prenatal diagnosis techniques has greatly increased the rate of prenatal diagnosis of fetal defects. The number of women with induced labor due to fetal congenital defects or stillbirth will be increasing year by year [25]. Termination of pregnancy can lead to severe posttraumatic stress disorder and strong psychological sadness response, which is common and lasting and may continue to affect the next pregnancy [26]. Giving appropriate psychological interventions before therapeutic induction of labor and during the puerperium can improve the patient's psychological well-being and build confidence to conceive again. At the same time, it is also conducive to promote the development of eugenics and the construction of mental health service system for this kind of population.

In this study, puerperal women carried out body relaxation and relaxation through yoga practice, so as to promote postpartum physical recovery, reduce the occurrence of postpartum complications, and alleviate the fear of poor postpartum physical recovery. It can help women better realize the meaning and self-value of life, improve the postpartum growth level of women with abnormal induced labor, and improve the quality of life. Previous studies have shown that 3-7 days after delivery are the peak period of anxiety and depression in puerperal women [27]. Compared to women with normal births, women with fetal abnormalities are 4 times more likely to suffer from depression, as well as 7 times more likely to suffer from PTSD. Intervention research on the psychological problems of women with fetal abnormalities in induced labor has also become a major topic in the world. The main psychological care intervention models include the provision of information support, supportive psychotherapy, grief counselling, and integrated clinical support services. The results indicated that after psychological nursing intervention, the scores of GAD-7, PHQ-9, IES-R, and LES were lower than those of routine nursing, while the score of NSNS was higher compared to routine nursing. The value of psychological care interventions in women with abnormal induction of labor has proved to be more remarkable. It is more helpful in reducing patients' anxiety and depression, improving the quality of life and increasing the satisfaction of care for women with abnormally induced labor. This is mainly due to the fear and worry of women who are induced with fetal abnormalities and their own low level of coping. In addition, these pregnant women do not have good control over the physical and emotional changes that occur during the puerperium. According to the psychological experience of puerperal women, we should formulate the theme of intervention, give positive guidance, and correct disease cognitive guidance to pregnant women. The disease-related information and emotional support should be provided, and postpartum continuous care should be supplied to support for women. It can help women better deal with fetal abnormal events, relieve anxiety and depression, and increase confidence in second pregnancy [28]. The earlier study found that relaxation training could increase the release of *α* brain waves and enkephalin in the human body to reduce the excitability of sympathetic nerve and relieve patients' negative emotions [29]. Sensible postnatal exercise can enhance a woman's sense of self-worth and self-confidence, thereby alleviating negative emotions. Postnatal exercise can also increase interpersonal and social resources and gain support from friends and/or family. This can reduce social isolation and therefore reduces the level of depression [30, 31]. This study still has some shortcomings. Firstly, the quality of this study is limited due to the small sample size we included in the study. Secondly, this research is a single-center study, and our findings are subject to some degree of bias. Therefore, our results may differ from those of large-scale multicenter studies from other academic institutes. This research is still clinically significant, and further in-depth investigations will be carried out in the future.

To sum up, the value of psychological care interventions in women with abnormally induced labor is more remarkable, contributing to the reduction of anxiety and depression and increasing the satisfaction of care for women with abnormally induced labor.

## Figures and Tables

**Figure 1:** Technology roadmap.

**Table 1:** The general data of two groups.

Group	Age (years)	Gestational week (week)	Educational level		Bad pregnancy history		With or without children		Type of conception		Fetal abnormality type	
			Senior high school and below (example/%)	Senior high school or above (example/%)	Yes (example/%)	None (example/%)	Yes (example/%)	None (example/%)	Natural conception (example/%)	Involuntary pregnancy (example/%)	Fetal malformation (case/%)	Stillbirth (example/%)
C group (*n* = 40)	31.15 ± 2.33	25.69 ± 3.19	20/50.00	20/50.00	20/50.00	20/50.00	17/42.50	23/57.50	20/50.00	20/50.00	17/42.50	23/57.50
R group (*n* = 40)	31.48 ± 2.16	25.74 ± 3.12	18/45.00	22/55.00	18/45.00	22/55.00	16/40.00	24/60.00	18/45.00	22/55.00	16/40.00	24/60.00
*t*/*χ*^2^	0.657	0.071	0.201		0.201		0.052		0.201		0.052	
*P*	0.513	0.944	0.654		0.654		0.820		0.654		0.820	

**Table 2:** The scores of GAD-7 before nursing and 4 weeks after discharge.

Grouping	Before nursing (points)	4 weeks after discharge (points)
Control group	15.28 ± 3.44	9.15 ± 2.27^∗^
Research group	15.31 ± 3.37	5.19 ± 1.04^∗^
*t* value	0.039	10.030
*P* value	0.968	<0.01

Note: ^∗^ represents the comparison before nursing and 4 weeks after discharge in this group, *P* < 0.05.

**Table 3:** The score of the PHQ-9 scale before nursing and 4 weeks after discharge.

Grouping	Before nursing (points)	4 weeks after discharge (points)
Control group	16.38 ± 3.23	8.77 ± 2.32^∗^
Research group	16.41 ± 3.21	5.72 ± 1.12^∗^
*t* value	0.041	7.487
*P* value	0.966	<0.01

Note: ^∗^ represents the comparison before nursing and 4 weeks after discharge in this group, *P* < 0.05.

**Table 4:** The score of the IES-R scale before nursing and 4 weeks after discharge.

Grouping	Before nursing (points)	4 weeks after discharge (points)
Control group	67.12 ± 7.39	47.29 ± 5.15^∗^
Research group	66.14 ± 7.27	28.25 ± 2.14^∗^
*t* value	0.597	21.592
*P* value	0.551	<0.01

Note: ^∗^ represents the comparison before nursing and 4 weeks after discharge in this group, *P* < 0.05.

**Table 5:** LES score before nursing and 4 weeks after discharge from hospital.

Grouping	Before nursing (points)	4 weeks after discharge (points)
Control group	78.59 ± 9.17	57.18 ± 5.39^∗^
Research group	78.63 ± 9.14	31.53 ± 3.11^∗^
*t* value	0.019	26.069
*P* value	0.985	<0.01

Note: ^∗^ represents the comparison before nursing and 4 weeks after discharge in this group, *P* < 0.05.

**Table 6:** The score of the NSNS scale before nursing and 4 weeks after discharge.

Grouping	Before nursing (points)	4 weeks after discharge (points)
Control group	58.44 ± 1.44	81.59 ± 2.11^∗^
Research group	58.12 ± 1.41	90.15 ± 3.36^∗^
*t* value	1.004	13.645
*P* value	0.318	<0.01

Note: ^∗^ represents the comparison before nursing and 4 weeks after discharge in this group, *P* < 0.05.

## Data Availability

The datasets used and analyzed during the current study are available from the corresponding author upon reasonable request.
